# Research on Network Model of Dentate Gyrus Based on Bionics

**DOI:** 10.1155/2021/4609741

**Published:** 2021-12-06

**Authors:** Jin Zhang, Xiaoping Wei, Shiwen Zhang, Xin Niu, Guang Li, Tiantian Tian

**Affiliations:** ^1^School of Information Science and Engineering, Hunan Normal University, Changsha 410000, China; ^2^School of Computer and Communication Engineering, Changsha University of Science and Technology, Changsha 410114, China; ^3^Science and Technology on Parallel and Distributed Laboratory, College of Computer, National University of Defense Technology, Changsha 410000, China; ^4^College of Control Science and Engineering, Zhejiang University, Zhejiang 310058, China; ^5^School of Information Engineering, Zhengzhou University of Science and Technology, Zhengzhou 450000, China

## Abstract

As an important part of the brain, the dentate gyrus has an irreplaceable effect in the process of memory generation. Therefore, the study of the dentate gyrus model has important significance in the study of brain function. This paper, combined with the real anatomical structure of the dentate gyrus, is based on the existing calculation model for studying the pathological state of the dentate gyrus, a network model of dentate gyrus based on bionics. Then, a simulation experiment on the normal dentate gyrus model is performed on the NEURON platform, the output of each neuron in the model is observed, and a conclusion that the improved model can respond to stimuli, generate action potentials, and transmit them along with the neural network is made. At the same time, the output results are compared with the existing pathological models, and the characteristics of the stimulus response between neurons in the dentate gyrus under normal physiological conditions are obtained. Finally, according to the semiquantitative classification definition and quantitative classification definition of the small-world network, the model is analyzed, and it is concluded that the improved dentate gyrus network model has small-world characteristics. Therefore, the neurons in the improved dentate gyrus model are tightly connected and can simulate the real dentate gyrus to a certain extent.

## 1. Introduction

As one of the most complex and mysterious organs known, the study of the structure and function of the brain has attracted wide attention. Among the many brain functions, learning and memory are the important advanced brain functions. The hippocampus is a key structure for learning and memory in mammals. It is mainly composed of CA1, CA3, and the dentate gyrus. The dentate gyrus is the main part of the hippocampus structure [1] and fully participates in the memory and learning process of the brain. At the same time, the dentate gyrus is the main entrance for the hippocampus to accept external information and is also the preprocessor of information. The dentate gyrus can separate the neural representation of similar memory through different neural circuits to optimize memory storage and subsequent retrieval [2, 3]. The dentate gyrus can be separated by mode [4, 5] to minimize the interference on specific memory storage and retrieval [6], and the function of precise regulation of memory can be achieved by establishing the synaptic connection between specific cells [7]. The existence of dentate gyrus makes the generation of memory organized and has important significance in the process of information coding [8] and processing and learning memory. Therefore, when studying the mechanism of memory generation, the dentate gyrus is the primary research object. However, it is not easy and usually impossible to directly use experimental means to explore the physiological activities of the dentate gyrus. Therefore, the concept of constructing the dentate gyrus model combines the qualitative research of the experiment with the quantitative analysis of the model to simulate the real physiological structure of the dentate gyrus as realistically as possible, providing an effective method for analyzing the physiological characteristics of the dentate gyrus [9]. This paper proposes a biophysical realistic and anatomical dentate gyrus computational model to study the stimulation After input, the general physiological characteristics of each neuron in the dentate gyrus and how the neurons respond to and adjust to the stimulus.

In recent years, biophysical models have been favored by many researchers. This model not only considers the true cell morphology and synaptic characteristics of various types of cells but also considers the dynamic mechanism of various ion channels. Multicompartment models are usually used. The atrioventricular model divides a spatially continuous single neuron into discrete multiple atria, which are interconnected to describe the temporal and spatial changes of neurons as a whole. According to different research purposes, these compartment models have different emphases on their structure and connection. Researchers have constructed many different types of dentate gyrus models according to different research purposes. The dentate gyrus model established by Patton and McNaughton [10] is used for numerical simulation. The model contains two excitatory neurons (granular cells and moss cells) and four inhibitory neurons (basket cells, axon-axon cells, and GPP cells) and layer II neurons of the entorhinal cortex. The dentate gyrus network model constructed by Tateno et al. [11] consists of 9 granular cells, 9 inhibitory interneurons, and 3 moss cells. The model is small and the connections between neurons are relatively simple.

In addition, the construction of pathological models of the dentate gyrus is also very common, especially in the study of the relationship between the dentate gyrus and temporal lobe epilepsy. Many researchers combine the changes in cells and neural circuits observed under pathological conditions to study the dynamic activities of the dentate gyrus model under normal and pathological conditions through a series of simulation experiments, aiming to find that the pathological state of the dentate gyrus is in epilepsy.

Lytton et al. [12] built a dentate gyrus model to simulate how the abnormality (reorganization) of the neural circuit caused by the germination of mossy fibers in the dentate gyrus can lead to abnormal excitation of the neural circuit in the case of temporal lobe epilepsy. The dentate gyrus model constructed by Santhakumar et al. [13] simplified literature [10] connects granular cells and granular cells to construct a dentate gyrus model under pathological conditions, which is used to study the loss of moss cells and the loss of moss cells after seizures and head injuries. Mossy fiber germination has a role in the hyperexcitability of the dentate gyrus. Dyhrfjeld-Johnsen et al. [14] established a 1 : 1 ratio structural model of the dentate gyrus based on the model in literature [13]. In addition, a functional model was established according to a 20 : 1 ratio, and two models were used to study epileptic seizures. Schneider et al. [15] parallelized the 20:1 functional model in literature [14] and further expanded the model scale to complete a 1:1 simulation of the functional model.

The construction of models in literature [14, 15] is based on the topological network form dentate gyrus model of literature [13] as the basic unit. This basic unit selects four types of neurons that are dominant in number and have clear research results, not only consider the divergence and convergence of synapses of different types of neurons but also consider the actual distribution of axons. However, in a truly healthy dentate gyrus, there is no connection between granule cells and granule cells, so the dentate gyrus model constructed by Santhakumar cannot be used to simulate a healthy dentate gyrus. Based on the principle of bionics, combined with the real anatomical structure of the dentate gyrus, this paper will propose a model structure of the dentate gyrus in a healthy state based on the topological network model of the dentate gyrus.

In the following section, we first introduce the physiological structure of the dentate gyrus and the existing pathological models, and then, based on the existing dentate gyrus model under pathological conditions, this paper removes the diseased part of the dentate gyrus model and constructs a general model under normal physiological conditions. Besides, the model's stimulus response characteristics and small-world characteristics are explained based on simulation experiments. Finally, the thesis summarizes the work of the whole article and proposes the future direction.

## 2. Modified Dentate Gyrus Model

### 2.1. Dentate Gyrus

Histologically, the composition of the dentate gyrus is divided into three parts: molecular layer (ML), granular cell layer (GL), and polymorphic layer (PL).

Among them, the polymorphic layer is also called a phylum (layer (hilus)), as shown in Figure 1 (the figure is quoted from the literature [14]).

Eight types of neurons are clearly defined anatomically in the dentate gyrus, which are granular cells (GC), mossy cells (MC), basket cells (BC), axons-axon cells (AAC), molecular layer cells that project to the anterior penetrating pathway (MOPP), hilar cells that project axons into the anterior penetrating pathway (HIPP), hilar cells that project axons into the commissural/combined pathway (HICAP), and interneurons. Cells have specific hierarchical cells (IS). According to the special properties of neurotransmitters released by neurons, the position in the layered structure of the dentate gyrus, the morphological structure, and the existence of specific markers, the neurons in the dentate gyrus are divided into excitatory neurons and inhibitory neurons. The first two types of neurons are excitatory neurons, and the last six are inhibitory neurons.

From the perspective of stratification, the molecular layer of the dentate gyrus is mainly composed of the dendrites of granular cells and the fibers projected from the stellate cells in the entorhinal cortex. The granular cell layer is the main cell layer of the dentate gyrus, densely arranged with granular cells. The innermost layer is the polymorphic layer, with axons of granular cells (also called mossy fibers) and other interneurons. Granular cells are the main projection neurons of the dentate gyrus. Granular cells, as their name suggests, are cells with a small spherical cell body, about 10 *μ*m in diameter, and arranged in the granular cell layer with a thickness of 4–6 cells [16]. The dendrites of granular cells extend vertically from the granular cell layer into the molecular layer covering this layer and can establish synaptic connections with multiple areas, mainly receiving projections from the entorhinal cortex II layer. The axons of granular cells, namely, mossy fibers, have no myelin sheath and are generated from the bottom of the cell body, extending downward into the polymorphic layer, not only targeting some interneurons, such as basket cells, moss cells, and HIPP cells, but also coalescing fiber bundles. Leaving the polymorphic layer and extending to the stratum lucidum of CA3, it establishes a synaptic connection with the pyramidal cells of CA3, and the projection process of granule cells to CA3 is also the only way for the dentate gyrus to project to its outer brain area. In addition, other types of neurons only function through internal connections in the dentate gyrus. There is no interconnection between granular cells, and indirect interactions are achieved through connections with other types of cells in the dentate gyrus.

As shown in Table 1, based on a large number of research results, the number and connection of various types of neurons in the dentate gyrus are given [17]. The first column of the table gives the number of each type of neuron. It can be observed that the numbers of GC, MC, BC, and HIPP are dominant. The data in the middle of the table shows the value or range of the number of postsynaptic neurons (from the first row) that a presynaptic neuron (from the first column) can connect to. For example, a GC can be combined with 7–12 MCs to establish synaptic connections. One MC can establish synaptic connections with 30,000–35,000 GCs. “—” means that there is no connection between the two types of neurons.

### 2.2. Pathological Model

The topological network forms dentate gyrus model constructed by Santhakumar mainly studies the role of pathological phenomena of moss fiber germination and moss cell loss in the hyperexcitability of the dentate gyrus. In the model, two granular cells are randomly selected for each granular cell to connect to simulate the phenomenon of moss sprouting. Moss cells remove all their connections to simulate the loss of moss cells. For the neuron model in the network, the modeling work of a single neuron is mainly completed from three aspects: the structure and attributes of the compartment model, the setting of ion channels, and the definition of dendritic spines.

In the model, according to the anatomical structure of the dentate gyrus neurons, the four largest numbers of neurons are divided into different compartments. The cell body is seen as a cylindrical chamber, dividing the dendrites into many nodes with uniform diameter and membrane characteristics, and then these nodes form a chamber. The dendrites close to the cell body are called proximal dendrites, and the dendrites are called distal dendrites which are far away from the cell body. The dendrites and cell bodies of a GC are divided into 9. The dendrites and cell bodies of an MC/BC are divided into 17 compartments, and the dendrites and cell bodies of a HIPP are divided into 13 compartments. The atrioventricular structure of the four neurons in the model is shown in Figure 2.

The four types of neurons in the dentate gyrus model are connected according to their axon distribution, as shown in Table 2. Take MC to GC as an example. Divergence means that an MC can connect to 200 GCs near it. A postsynaptic target pool means that an MC chooses to connect among 350 GCs near it. Distribution characteristics, excluding the closest 50 GCs, convergence means that 6. 0 ± 0. 05 MCs can be connected to the same GC. “—“ means that there is no connection between the two types of neurons. In addition, the sprouting of moss fibers is simulated by adding connections between GCs, and the number of connections between GCs varies with the degree of sprouting.

### 2.3. Improvement of the Model

The existing topological network dentate gyrus model constructed by Santhakumar mainly simulates the pathological phenomenon of moss sprouting and MC loss caused by epileptic seizures or head injury and analyzes the influence of these two phenomena on the hyperexcitability of the dentate gyrus. Under normal physiological conditions, there is no connection between GCs, while under pathological conditions, the sprouting of moss cells leads to the formation of connections between GCs, and the number of connections formed varies with the degree of disease. GC interconnection leads to increased excitability of the network. The loss of MC reduces the number of model GC connections, hinders the spread of network hyperexcitability, and reduces the excitability of the model. The existing dentate gyrus model randomly selects GCs to form connections to simulate the phenomenon of moss sprouting when establishing connections for each GC and randomly selects several MCs and removes all their connections to simulate MC loss.

Compared with the existing dentate gyrus model, the dentate gyrus model proposed in this paper removes the connection between GCs that simulate mossy fiber sprouting, ensuring that GCs are not directly connected, and maintaining the normal connection between MCs to eliminate MC missing Therefore, the improved model can simulate the general dentate gyrus simulation model under normal physiological conditions as shown in Figures 3 and 4.

The connections between cells in the model conform to the connections between cells in the real dentate gyrus. The improved model has the following characteristics:

1. The first characteristic is covering the main neurons of the dentate gyrus.
2. There are four types of neurons in the dentate gyrus, GC, MC, BC, and HIPP, which dominate. Since the other four types of neurons have relatively few physiological data and cannot support the modeling needs, the model only contains four types of neurons: GC, MC, BC, and HIPP [3].
3. The number of neurons follows anatomical results.
4. From Table 1, the numbers of GC, MC, BC, and HIPP are 1 ^*∗*^ 106, 3 ^*∗*^ 104, 1 ^*∗*^ 104, and 1.2 ^*∗*^ 104, respectively. Therefore, in the improved dentate gyrus model, the ratio of the number of four types of neurons is GC: MC: BC: HIPP = 500: 15: 5: 6.
5. The third characteristic is a more complete simulation of the nerve pathways in the dentate gyrus.
6. According to the internal physiological anatomy of the dentate gyrus, GC is the main input neuron of the dentate gyrus. All GCs can be given input through the anterior penetrating pathway. At the same time, all BCs and 15% of MCs will also receive input from the entorhinal cortex. However, there is no direct connection between GCs, and indirect interconnection can be achieved through connections with other types of neurons. In addition, the model has rich internal connections. Except for the case where BC does not project to HIPP, there are interconnections between these four types of neurons, and MC and BC also have connections between neurons of the same type. GC is also the only output neuron in the dentate gyrus, which outputs information to CA3.

## 3. Experiment

Perform simulation experiments on the improved dentate gyrus model on the NEURON platform, and observe the output of each neuron in the model. In this process, only some parameters of the neuron need to be set, such as geometric shape, biophysical parameters, and connection relations, without considering the mathematical model used behind it and the complicated numerical solution process.

### 3.1. Simulation Platform

Modeling and simulation research can not only observe the changes of single-neuron activity and the simultaneous firing of neuron clusters but also examine the network connections and interactions between these neurons. Based on the structure, physiological characteristics, and biophysical principles of the above-mentioned dentate gyrus, this paper uses NEURON software to simulate the improved dentate gyrus model.

NEURON software was developed by researchers from Duke University and Yale University. It is a simulation environment for modeling individual neurons and neural networks. After iterative optimization, it has become the most popular neural modeling tool in the world. The specific modeling process is shown in Figure 5. NEURON software provides some tools that can conveniently construct, manage, and use models in a reasonable and computationally efficient manner. It is especially suitable for problems closely related to experimental data, especially those involving nerves with complex anatomical and biophysical characteristics.

NEURON software provides two methods for building neural system models. The first is the graphical user interface (GUI), which does not require any programming code, such as CellBuilder (create neuron model), Channel Builder (build ion channel model), Linear Circuit Builder (linear neural circuit generator), and NetWork Builder (to build a small network prototype). The second is to use HOC language to write custom model parameters to achieve more complex functions.

NEURON software includes two programming languages, namely, high-level calculation language (High Order Calculator (HOC) and Model Description Language (NMODL)). Using GUI to construct neural system model description parameters such as morphology and characteristics is relative. It may not meet the actual complex network construction. HOC language implements some of the features of object-oriented programming and has a large number of built-in library functions, allowing users to customize complex network models. NMODL language is mainly used to describe neuron cell membranes. The NEURON software also embeds ready-made ion channel models and synaptic connection models. These models can be directly called and set through GUI or HOC language. Of course, various electrophysiological characteristics can also be customized through NMODL, such as the calcium ion channel model and potassium ion channel model.

The advantages of NEURON software can be divided into the following aspects:

1. The basic model function library of biophysics is embedded. The more commonly used of these models are the H-H equation and the synaptic connection equation (EXP). The user only needs to call these functions to build the model and observe the overall characteristics of the model without considering the complicated numerical solution process involved in the middle. This is also one of the design goals of the NEURON software, helping modelers solve advanced neuroscience research problems, without being bothered by low-level math or calculation problems.
2. Provide a variety of numerical integration methods. The reverse Euler method is a basic numerical integration method. It is relatively simple and has good stability. Although the accuracy is not high enough, it can still meet most of the needs. The Crank–Nicolson method has higher accuracy and stability, but it takes more time. The adaptive integration method can flexibly adjust the order and step length according to the actual situation and has achieved the goal of fast and high precision.
3. GUI simplifies the difficulty of model construction. You can set parameters directly on the GUI, create a single neuron model or a nervous system model composed of multiple neuron models, and control the simulation process to view the output of the model.

However, in the modeling process, the new hoc language of the NEURON platform has increased the difficulty of modeling, and there are fewer books and related materials that can be referred to and learned; at the same time, because of the content of biological neural networks involved in our NEURON programming, if the understanding is not deep, it is somewhat difficult to explain the accidental phenomena in the experiment. But on the basis of the existing model, we have a new understanding and a deeper understanding of NEURON modeling, which provides us with great help.

### 3.2. Simulation Experiment

A simulation model is established based on the NEURON simulation platform, and the stimulus introduced by a single artificially stimulated cell is used as input. Among them, 100 GCs, 2 BCs, and 2 randomly selected MCs to receive stimulation, which is equivalent to the actual dentate gyrus nervous system through perforation. The stimulus of path transmission. The NetStim class transmits a single stimulus, and the custom VecStim class generates continuous stimuli by reading the time of the input pulse in the file. The model saves the network connection and the point changes of the gods in the file through the file interface and displays the image of the neuron potential change and the image of the network activity.

Set the time step of numerical calculation to 0.1 ms and the duration to 100 ms and 5 ms after the start of the simulation, provide an input stimulus for the model, with the duration of the simulation as the horizontal axis, in milliseconds, and the membrane potential as the vertical axis, in millivolts, and observe the changes in neuron potential. When there is no external stimulus, the neuron is resting. Under normal circumstances, the resting potential of the neuron is usually around −70 mV; when the cell membrane is stimulated, a potential change occurs. When the membrane potential reaches a threshold of around −40 mV, the original negative potential in the membrane disappears quickly, the potential becomes 20 mV to 40 mV, and the amplitude of the entire membrane potential change can reach 90 to 130 mV. The resting potentials, action potentials, and thresholds of neurons in the model are shown in Table 3. The changes of the membrane potentials of the four types of neurons are in line with the general rules of neuron action potentials.

The time for each neuron in the improved model to receive stimulation, reach the threshold, appear peak, and return to rest is in Table 4. The input stimulation time of artificially stimulated neurons in the 5^th^ ms. Due to the cell delay, transmission delay, and synaptic delay in the network, the GC, BC, and MC receiving stimulation time has a delay of about 4 ms. For HIPP and unstimulated HIPP, because MC does not accept external stimuli, the time of generating action potentials is later than that of neurons directly receiving input stimuli.

Perform simple simulation experiments on the improved dentate gyrus model on the NEURON simulation platform. First, based on the number of neurons and electrophysiological data, only the four types of neurons in the dentate gyrus that have an absolute advantage in number are modeled. These four types of neurons are granular cells (GC) and moss cells (MC), Basket cells (BC), and HIPP cells. According to the number of these four main types of neurons, a reduction ratio of 2,000 : 1 is used to construct a simplified simulation model of the dentate gyrus. The proportion of the number of the four kinds of neurons after reduction was GC: MC: BC: HIPP = 500:15:5:6.

In the simulation experiment, the time step of the numerical calculation is set to 0.1 ms and the duration is 100 ms. Before the stimulation is introduced, the membrane potential of each neuron is set to the resting potential of −60 mV. 5 ms after the start of the simulation, an input stimulus is provided to the model. At this time, the simulation model uses the stimulus introduced by a single artificial stimulation cell as input. Then, the model saves the network connection and the point changes of the gods in the file through the file interface and displays the image of the neuron potential change. In the displayed potential change image, the simulation duration is taken as the horizontal axis and the unit is milliseconds, and the membrane potential is taken as the vertical axis and the unit is millivolt; observe the changes in neuron membrane potential.

Figure 6 shows the comparison of the neuron potential diagram and the network activity diagram before and after the model is improved. Figures 6(a) and 6(b) are the network activity diagrams before and after the model is improved, and Figures 6(c) and 6(d) are the neuron potential changes before and after the model is improved. Comparing Figures 6(a) and 6(b) and Figures 6(c) and 6(d), it can be seen that removing the connection between GCs in the model reduces the excitability of the model and the stimulation transmission between neurons in the model. This phenomenon is consistent with the physiological characteristics of reduced excitability of the dentate gyrus after removing the pathological state of mossy fiber sprouting. When the stimulus is transmitted inside the model, there is a significant difference in the changes of the cell body potential of MC and BC in the model before and after the improvement. The potential changes of BC before and after the model is improved are shown in Figure 6(e). Before the model is improved, BC will not only receive stimulation from artificially stimulated neurons. After about 10 ms, the stimulus transmitted through the neural network generates an action potential. After the model is improved, the excitability of the model is reduced. Only the input stimulus makes the BC produce action potentials, and there is no stimulus from the network.  Figure 6(f) shows the change of MC cell body potential before and after model improvement. MC only accepts input stimulation. It can be seen from the figure that due to the delay of synaptic and axon conduction in the network, the action potential is generated late. Therefore, the improved model can simulate the dentate gyrus in a healthy state to a certain extent.

It can be seen from the figure that the time, peak value, and number of action potentials generated by the four types of neurons are different, and the time to restore resting potentials is also different. In the real biological nervous system, different types of neurons have different characteristics and different stimulus transmission distances, and there will also be delays, such as cell delays, transmission delays, and synaptic delays [18]. In addition, to analyze the stimulus response characteristics of the improved neurons more clearly, the same neuron's different position membrane potential changes were also observed. It is known from the 2^nd^ section that each GC is provided with two dendrites, and each dendritic is divided into four sections, namely, four compartments. According to the distance between the dendrites and the cell body, mark the first section, the second section, the third section, and the fourth section from the near and far, respectively, and then record the potential change of the dendrites in each section.

Figures 7–10 show the changes in the membrane potential of the first GC dendrites at different positions, from the distal dendrites of the GC (the fourth section) to the proximal dendrites (the first section) and then to the cell body; the peak value of the membrane potential gradually increases. After inputting the stimulation, different neurons in the model and different positions of the same neuron respond quickly to generate action potentials. After the stimulation, they gradually return to a stable state. This phenomenon is consistent with the stimulation-response characteristics of real neurons. The experimental results show that the improved dentate gyrus model can respond to stimuli like real neuron networks, generate action potentials, and transmit the stimuli along with the neural network.

### 3.3. Analysis of Small-World Characteristics

The biological nervous system is a typical complex network, and its network structure can be understood through anatomical knowledge. However, in most research situations, you want to understand some of the hidden characteristics behind the structure of the nervous system. At this time, you need to use relevant analysis tools for research. Graph theory is usually used to analyze the biological nervous system. Neurons are represented as graph nodes, and the connections between neurons are represented as edges of the graph. This equivalent diagram is analogous to the connection mode of the nervous system, and then some characteristics contained in the equivalent diagram are studied. Among them, the small-world network theory is very suitable for studying highly clustered, tightly interconnected sparse networks.

To better study the topological characteristics of network structure, Watts and Strogatz [19] proposed and mathematically defined the concept of a small-world network. In this kind of network, there are two key indicators: the average distance between nodes L and the clustering coefficient C. The average distance between nodes L reflects global connectivity, and it is defined as follows. Suppose there is a graph G with N nodes; the shortest path length d between two nodes represents the least number of edges passed in the process from one node to another. Formula (1) represents the average path length of node *i*, and formula (2) shows the average path length of the network. The clustering coefficient *C* is used to indicate the degree of local connectivity of the network. A node with k neighbors can have at most *k*(*k* − 1)/2 edges. First, calculate the ratio of the actual number of edges between each node and the neighbor *E* to *k*(*k* − 1)/2, and then calculate the average of the ratios of all nodes as the clustering coefficient *C*. Equation (3) represents the clustering coefficient of node *i*, and (4) represents the clustering coefficient of the network. The clustering coefficient *C* is a coefficient describing the degree of aggregation between nodes in the network and represents the degree of connection between adjacent nodes of a node in the network:

(1) $$\begin{array}{c} L_{i}=\frac{\sum_{i>j>0}^{N}d_{ij}}{N-1}, \end{array}$$

(2) $$\begin{array}{c} L=\frac{1}{N}\sum_{i=1}^{N}L_{i}, \end{array}$$

(3) $$\begin{array}{c} C_{i}=\frac{2E_{i}}{k_{i}\left(k_{i}-1\right)}, \end{array}$$

(4) $$\begin{array}{c} C=\frac{1}{N}\sum_{i=1}^{N}C_{i}. \end{array}$$

Generally speaking, the network topology can be divided into three types: (1) regular network (regular network), where the distance between any two connected nodes is the closest, and the two nodes that are farther apart are separated by a large number of nodes in the middle, and *L* and *C* are both large; (2) random network (random network), contrary to regular network, the connection of each node is not restricted by space, *L* and *C* are both small; (3) small-world network, the global connectivity of its nodes And local connectivity is between the other two types of networks. There are connections with neighboring nodes and connections with distant nodes; in other words, if *L* is small, *C* is large.

When judging whether a network has the characteristics of a small world, it cannot be judged directly based on the size of *L* and *C*. Usually, first find out the equivalent random graph corresponding to the network. The number of nodes, the number of edges, and the average degree of the random graph are the same as those of the network 〈*k*〉 and calculate *L*_rand_ and *C*_rand_; see (5) and (6). If *L* ≥ *L*_rand_ and *C* >> *C*_rand_, it means that the network has small-world characteristics. This judgment method is called the semiquantitative categorical definition of the small-world network [18]:

(5) $$\begin{array}{c} L_{\text{rand}}=\frac{\ln\;N}{\ln\langle k\rangle }, \end{array}$$

(6) $$\begin{array}{c} C_{\text{rand}}=\frac{\langle k\rangle }{N}. \end{array}$$

Then, the small-world quotient *Q* is introduced to represent the characteristic parameters of the small-world characteristics. The formula is shown in (7). If the small-world quotient *Q* is greater than 1, it means that the network has small-world characteristics. The larger the quotient *Q*, the more obvious the small-world characteristics of the network [20]:

(7) $$\begin{array}{c} Q=\frac{C/L}{C_{\text{rand}}/L_{\text{rand}}}. \end{array}$$

After the simulation experiment is over, the connection matrix of the improved model can be obtained. Then, calculate *C* and *L*, as well as *C*_rand_ and *L*_rand_ graphs of equivalent random numbers. The calculation results are in Tables 5 and 6.

From the calculation results in Tables 5 and 6, *L* < *L*_rand_, and a smaller L indicates that, on average, the improved dentate gyrus model maintains a good relationship in the global scope. *C* >> *C*_rand_, in line with the high clustering coefficient of the small-world network. From the small-world quotient *Q* > 1, it shows that the improved dentate gyrus model has small-world characteristics. At the same time, the small-world quotient of the improved model is greater than the small-world quotient of the model before the improvement, indicating that the small-world characteristics of the improved model are more obvious than those before the improvement. This shows that the improved dentate gyrus network model can simulate the real neural network to a certain extent, and combined with the bionic experiment results of the improved model on the NEURON platform, this paper can conclude that the improved bionic model can simulate to a certain extent True healthy dentate gyrus.

## 4. Conclusions

Based on the research of the pathological dentate gyrus model constructed by Santhakumar, this paper proposes an improved dentate gyrus model and conducts simulation experiments and structural analysis. This paper first introduces the structure, neurons, and connections of the dentate gyrus in detail, as well as an existing model of the dentate gyrus under pathological state. Then, based on the idea of bionics, the dentate gyrus model was improved, following the connection of healthy dentate gyrus neurons as much as possible under real conditions, and deleting the connection between granular cells and granular cells. Then, the simulation of the model is completed on the NEURON platform. From the changes in membrane potential, the neurons in the model can respond to the input stimulus to generate action potentials and transmit the stimuli, which conforms to the physiological characteristics of neurons. Finally, the definition of the small-world network is used to judge the small-world characteristics of the improved model. Through the analysis of the experimental results, the improved dentate gyrus model truly simulates the connections between dentate gyrus neurons to a certain extent.

The improved model becomes more realistic and versatile, can better describe the functional role of cell types in the dentate gyrus, and is of great significance for subsequent functional studies of the dentate gyrus. By modeling the dentate gyrus in a healthy state, it can analyze its physiological characteristics more clearly, which is of reference significance for clinical research on diseases caused by the dentate gyrus. In the future, it will be considered to combine the model with the field of deep learning [21] and the medical knowledge map [22] to improve the model's bionic degree and expand the application range of the model.

## Figures and Tables

**Figure 1:** Cell types and connections of the dentate gyrus [14].

**Figure 2:** Improved cell connection of dentate gyrus model.

**Figure 3:** Improved topological structure of dentate gyrus network model.

**Figure 4:** Improved cell connection of dentate gyrus model.

**Figure 5:** The specific process of modeling with NEURON.

**Figure 6:** Comparison of neuron potential diagram and the network activity diagram before and after model improvement. (a) Image of neuron activity before model improvement. (b) Neuron activity image after model improvement. (c) Change curve of neuron cell body potential before model improvement. (d) Change curve of neuron cell body potential after model improvement. (e) Comparison of BC cell body potential changes before and after model improvement. (f) Comparison of MC cell body potential changes before and after model improvement.

**Figure 7:** Changes of membrane potential in the middle position of the dendrites in the fourth section of the first GC.

**Figure 8:** Changes of membrane potential in the middle position of the dendrites in the third section of the first GC.

**Figure 9:** The change of membrane potential in the middle of the dendrites of the second node of the first GC.

**Figure 10:** The change of membrane potential in the middle of the dendrites of the first section of the first GC.

**Table 1:** Connection phenomena of dentate gyrus cells [16].

	GC	MC	BC	AAC	MOPP	HIPP	HICAP	IS
GC (1,000,000)	—	7–12	10–20	1–5	—	100–120	30–50	10–30
MC (30,000)	30,000–35,000	200–500	5–10	5–10	5	600	200	—
BC (10,000)	1,000–1,500	50–100	20–50	—	—	0–1	—	—
AAC (2,000)	2,000–4,000	100–200	—	—	—	—	—	—
MOPP (4,000)	5,000–10,000	—	30–50	1–2	5–10	—	5–10	—
HIPP (12,000)	1,500–1,600	20–50	400–500	20–40	10–20	—	10–20	—
HICAP (3,000)	700	30–40	150–200	—	10–20	50	50	—
IS (3,000)	—	—	5–10	—	—	5–10	5–10	100–800

**Table 2:** Model connection parameters [13].

	From (column)/to (row)	GC	MC	BC	HIPP
GC	Divergence	Sprouted	1:1	1:1	1:1
	Topographic postsynaptic target pool	100	3	3	5
	Convergence	Varied with sprouting	33 ± 0.09	83.33 ± 2.26	250 ± 6.7

MC	Divergence	1:200	1:3	1:1	1:2
	Topographic postsynaptic target pool	350 (except 50 in the center)	6	3 (except 1 in the center)	5
	Convergence	6.0 ± 0.05	3.0 ± 0.3	2.5 ± 0.5	5.0 ± 0.5

BC	Divergence	1:100	1:3	1:2	—
	Topographic postsynaptic target pool	140	7	3	—
	Convergence	1.2 ± 0.03	1.2 ± 0.24	2 ± 0.36	—

HIPP	Divergence	1:160	1:4	1:4	—
	Topographic postsynaptic target pool	260	5	5	—
	Convergence	1.92 ± 0.03	1.6 ± 0.16	4.0 ± 0.45	—

**Table 3:** Changes in membrane potential of four types of neurons in experimental models.

Model potential	GC	MC	BC	HIPP
Model resting potential (mV)	−70.44	−60.11	−60	−70.67

Peak model action potential (mV)	37.14	46.72	46.87 (5.58)	76.53

Model threshold (mV)	−39.44	−39.05	−38.86	−42.67

**Table 4:** The change time of each neuron potential in the simulation experiment model.

Time	G cell	B cell	M cell	H cell
Stimulation time (ms)	9.0	9.4	8.9 (15.7)	15.6
Time to threshold (ms)	13.6	12.9	13.4 (30.9)	16.9
Time to peak (ms)	14.0	13.4 (16.5)	14.10 (32.0)	17.3
Rest time (ms)	76.0	55.5	37.4 (52.6)	35.5

**Table 5:** Small-world characteristics statistics before model improvement.

〈*k*〉	*L*	*C*	*L*_rand_	*C*_rand_	*Q*
46.4061	2.0919	0.2074	2.3015	0.0428	5.3313

**Table 6:** Small-world characteristic statistics of the improved model.

〈*k*〉	*L*	*C*	*L*_rand_	*C*_rand_	*Q*
27.4118	2.1273	0.2092	2.6745	0.0252	10.1943

## Data Availability

The experimental data required in the article has been described in detail in the article (visit https://github.com/weniu/Dentate-gyrus-NEURON).

## Additional Points

CCS concepts include computing methodologies, modeling and simulation, model development and analysis, and model verification and validation.
